The article "Preoperative Predictors of Optimal Tumor Resectability in Patients With Epithelial Ovarian Cancer" was published in 2022. Journal: Cureus.

# Preoperative Predictors of Optimal Tumor Resectability in Patients With Epithelial Ovarian Cancer

**DOI:** 10.7759/cureus.21409

**Published:** 2022-01-19

**Authors:** Kehinde S Okunade, Adaiah P Soibi-Harry, Benedetto Osunwusi, Ephraim Ohazurike, Sarah O John-olabode, Adeyemi Okunowo, Garba Rimi, Omolola Salako, Muisi Adenekan, Rose Anorlu

**Affiliations:** 1 Obstetrics and Gynaecology, Lagos University Teaching Hospital, Lagos, NGA; 2 Obstetrics and Gynaecology, College of Medicine, University of Lagos, Lagos, NGA; 3 Haematology, College of Medicine, University of Lagos, Lagos, NGA; 4 Obstetrics and Gynaecology, College of Medicine, University of Lagos/Lagos University Teaching Hospital, Lagos, NGA; 5 Radiotherapy, Lagos University Teaching Hospital, Lagos, NGA

**Keywords:** primary debulking surgery, eoc, optimal tumor resectability, lagos, otr, ovarian cancer

## Abstract

Background

Several studies have shown that whether complete tumor resection can be achieved during debulking surgery depends on various patient-related factors. However, none of these studies was conducted among patients with epithelial ovarian cancer (EOC) in sub-Saharan Africa. In this study, we aimed to determine the preoperative predictors of optimal tumor resectability (OTR) during primary debulking surgery (PDS) in patients with EOC.

Methodology

In this study, we reviewed all patients with histologically diagnosed EOC who underwent PDS between January 2011 and December 2020. We included 83 patients with complete clinical records for subsequent data analysis. Descriptive statistics were computed for patients’ data, and binary logistic regression analysis was used to assess the strength of associations between patients’ preoperative characteristics and OTR.

Results

The overall rate of OTR was 53.0%, while the rate in advanced EOC patients was 36.1%. In the univariate analyses, pleural effusion, ascites, tumor bilaterality, size of the largest tumor, retroperitoneal lymph nodes, omental caking, peritoneal thickening, significant extrapelvic tumor, serum cancer antigen-125 (CA-125) levels, and hemoglobin levels were recorded as the predictors of OTR. However, after adjusting for covariates in the final multivariate models, we found that the absence of moderate-to-large pleural effusion (odds ratio (OR) = 5.60; 95% confidence interval (CI) = 1.32, 23.71) and having serum CA-125 levels of ≤370 U/mL (OR = 6.80; 95% CI = 1.19, 38.79) were the overall independent predictors of OTR while not having any preexisting comorbidity (OR = 18.21; 95% CI = 2.40, 38.10), and the absence of pleural effusions (OR = 13.75; 95% CI = 1.80, 24.85) or enlarged retroperitoneal lymph nodes (OR = 11.95; 95% CI = 1.35, 16.07) were predictors of OTR in advanced EOC patients.

The article "Preoperative Predictors of Optimal Tumor Resectability in Patients With Epithelial Ovarian Cancer" was published in 2022. Journal: Cureus.

Conclusions

We demonstrated that the radiological absence of pleural effusions and enlarged retroperitoneal lymph nodes and having no preexisting medical morbidity and serum CA-125 levels of ≤370 U/mL were the independent predictors of OTR during PDS. The preliminary data generated from this study can be used to develop variables for a prediction model in a future validation study.

## Introduction

In Nigeria, ovarian cancer (OC) is the second most common gynecologic cancer [1,2], with a peak incidence among women in their early 60s [2]. Approximately 90% of all histological types of OC are epithelial in origin [3], with over 70% of cases diagnosed at an advanced stage (International Federation of Gynecology and Obstetrics (FIGO), stage III-IV) [2]. Patients with epithelial ovarian cancer (EOC) are conventionally treated by primary debulking surgery (PDS) followed by adjuvant platinum-based chemotherapy [4]. One of the most important predictors of survival in patients with advanced EOC is the size of residual tumor after PDS [5]. Therefore, the goal of primary surgery is to achieve optimal tumor resectability (OTR). OTR is achieved when the residual tumor after surgery is less than 1 cm in the largest diameter [6]. Patients with advanced FIGO stage of EOC may undergo extensive debulking surgery and still have a significant residual tumor with a subsequent poor oncologic outcome and ultimate reduction in overall survival [2]. Therefore, patients with a low probability of optimal primary surgical debulking have the option of undergoing neoadjuvant chemotherapy (NACT) followed by interval debulking surgery to increase their chances of optimal surgical outcomes and subsequent improvement in survival [7,8].

Whether OTR can be achieved during debulking surgery depends on various patient factors such as age, comorbidity, extent, and location of the disease, as well as the skill and experience of the operating surgeon [9,10]. Therefore, it is important to develop an algorithm using these various preoperative factors derived from patient-specific characteristics and radiologic findings to predict patients with advanced EOC who may benefit from upfront or PDS. This study was aimed to determine the preoperative clinical and radiologic predictors of OTR during PDS in patients with EOC in Lagos, Nigeria.

## Materials and methods

Study design

We conducted a review of the health records of all OC cases that were managed at a university teaching hospital in Lagos, Nigeria between January 2011 and December 2020.

Study setting

This study was conducted at a foremost public tertiary health institution in Lagos that offers specialized care including gynecologic oncology services. The hospital is the main referral center for other government-owned and private hospitals in Lagos and its neighboring states. Lagos State is the commercial capital of Nigeria with a population of 20 million [2].

The article "Preoperative Predictors of Optimal Tumor Resectability in Patients With Epithelial Ovarian Cancer" was published in 2022. Journal: Cureus.

Eligibility criteria

We included 83 patients with histologically diagnosed EOC who underwent PDS during the review period. Women with non-epithelial OC, those who underwent NACT before debulking surgery, and those without complete clinical records or relevant data for analysis were excluded.

Data collection

Data retrieved from patients’ medical records included age, parity, menopausal status, body mass index (BMI), serum cancer antigen-125 (CA-125) levels, coexisting morbidity (such as hypertension, diabetes mellitus, kidney, and liver disease), presence of pleural effusion (on chest X-ray or chest computed tomography (CT) scan), ascites, tumor bilaterality, largest tumor diameter, the presence of retroperitoneal lymph nodes, omental caking (metastasis), peritoneal thickening and significant extrapelvic tumor with size greater than 2 cm on radiological imaging using abdominopelvic ultrasound and/or CT scan, and the outcome of PDS (optimal/suboptimal).

Study endpoints

The study endpoints included (1) the rate of OTR, and (2) the preoperative predictors of OTR during PDS in patients with EOC. OTR is achieved when the residual tumor after PDS is less than 1 cm in the largest diameter [6].

Statistical analysis

Data analysis was performed using SPSS version 27.0 (IBM Corp., Armonk, NY, USA), and descriptive statistics were computed for all patients’ baseline characteristics. Patient characteristics were described using mean and standard deviation (if normally distributed) or median and interquartile range (if skewed) for continuous variables and by frequencies and percentages for categorical variables. Binary logistic regression models were used to estimate the odds ratios (ORs) and 95% confidence interval (CIs) for baseline demographic and clinical characteristics of patients. Adjustments were made to include factors with P < 0.10 in the final multivariate models. Associations were considered statistically significant if P-values were <0.05.

Ethical considerations

We obtained ethical approval from the Health Research Ethics committee of the Lagos University Teaching Hospital (ADM/DCST/HREC/1912) before retrieving medical records and data collection. We conducted the study following the ethical principles of the Helsinki Declaration.

## Results

A total of 156 cases of OC were managed in the hospital during the period under review, of which 83 were eligible for inclusion in the final analysis. We excluded 18 women with non-EOC histotypes, 46 who had neoadjuvant chemotherapy and interval debulking surgery (NACT+IDS), five who failed to undergo treatment, and four with insufficient clinical data for analysis (Figure 1).

The article "Preoperative Predictors of Optimal Tumor Resectability in Patients With Epithelial Ovarian Cancer" was published in 2022. Journal: Cureus.

**Figure 1:** Patient selection chart. EOC: epithelial ovarian cancer; NACT: neoadjuvant chemotherapy; IDS: interval debulking surgery

The mean age of the patients in the study group was 54.5 ± 11.5 years. Patients were predominantly in the 50-59-year age group (n = 28, 33.7%), multiparous (n = 53, 63.8%), postmenopausal (n = 45, 54.2%), and had normal BMI (n = 37, 44.6%). More than two-thirds of the patients had coexisting medical morbidities (n = 64, 77.1%) and approximately half (n = 41, 49.4%) had significant ascites on radiological imaging (Table 1). Pleural effusions were seen in over two-thirds (n = 57, 68.7%) of the patients, while less than one-fifth had retroperitoneal lymphadenopathy (n = 16, 19.3%). Less than half of the patients (n = 35, 42.2%) had a bilateral tumor, with about one-third (n = 26, 31.3%) having omental metastasis. Peritoneal thickening (n = 33, 39.8%) and significant extrapelvic tumor greater than 2 cm (n = 36, 43.4%) were detected in approximately two-fifths of EOC patients. The median tumor size on radiological imaging and the median levels of other hematologic markers are presented in Table 1.

**Table 1:** Characteristics of patients with epithelial ovarian cancer (n = 83). BMI: body mass index; CA-125: cancer antigen-125; IQR: interquartile range; SD: standard deviation

Characteristics	Number (%)
Mean age, years (±SD)	54.4 ± 11.5
20–29	1 (1.2)
30–39	11 (13.3)
40–49	17 (20.5)
50–59	28 (33.7)
60–69	14 (16.9)
≥70	12 (14.5)
Median parity (IQR)	2 (1–3)
<2	30 (36.1)
2–5	48 (57.8)
>5	5 (6.0)
Menopausal status	
Premenopause	38 (45.8)
Postmenopause	45 (54.2)
Coexisting morbidity	
Yes	19 (22.9)
No	64 (77.1)
Mean BMI, kg/m^2 ^(±SD)	26.0 ± 4.8
Underweight <18.5	2 (2.4)
Normal weight 18.5–24.9	37 (44.6)
Overweight 25–29	26 (31.3)
Obese ≥30	18 (21.7)
Pleural effusions	
Yes	26 (31.3)
No	57 (68.7)
Ascites	
Yes	41 (49.4)
No	42 (50.6)
Tumor bilaterality	
Bilateral	35 (42.2)
Unilateral	48 (57.8)
Retroperitoneal lymph nodes	
Absent	67 (80.7)
Present	16 (19.3)
Omental cakeing	
Yes	26 (31.3)
No	57 (68.7)
Peritoneal thickening	
Yes	33 (39.8)
No	50 (60.2)
Extrapelvic tumor >2 cm	
Yes	36 (43.4)
No	47 (56.6)
Median largest tumor size, mm (IQR)	59 (43–88)
Median serum CA-125 levels, U/mL (IQR)	370 (144–675)
Median hemoglobin levels, g/dL (IQR)	10.5 (9.4–11.4)
Median white cells count, ×10^9^/L (IQR)	6.5 (4.8–8.8)
Median platelet count, ×10^9^/L (IQR)	333 (203–427)

The overall rate of OTR in this study was 53.0%, while the rate among EOC patients with advanced (FIGO stage III and IV) disease was 36.1%. As shown in the univariate analyses (Table 2), the absence of radiologically visible pleural effusion (P = 0.006), ascites (P = 0.003), retroperitoneal lymph nodes (P = 0.012), omental caking (P = 0.003), peritoneal thickening (P = 0.001), and significant extrapelvic tumor (P = 0.001) together with unilateral ovarian tumor (P = 0.001), largest tumor diameter <60 mm (P = 0.037), serum CA-125 levels of ≤370 U/mL (P = 0.001), and hemoglobin levels of ≤10.5 g/dL (P = 0.096) were the likely predictors of OTR during PDS. However, after adjustments in the final multivariate models (Table 3), having no comorbidity and serum CA-125 levels of ≤370 U/mL (OR = 6.80; 95% CI = 1.19, 38.79; P = 0.031) and the absence of any radiological evidence of pleural effusions (OR = 5.60; 95% CI = 1.32, 23.71; P = 0.019) and enlarged retroperitoneal lymph nodes were the only independent predictors of optimal PDS.

The article "Preoperative Predictors of Optimal Tumor Resectability in Patients With Epithelial Ovarian Cancer" was published in 2022. Journal: Cureus.

**Table 2:** Univariate analyses of preoperative predictors of surgical outcomes in epithelial ovarian cancer (n = 83). BMI: body mass index; CA-125: cancer antigen-125; CI: confidence interval; OR: odds ratio

Characteristics	Surgical resectability		Unadjusted OR (95% CI)	P-value
	Optimal n = 44 (%)	Suboptimal n = 39 (%)		
Coexisting morbidity				0.627
No	33 (75.0)	31 (79.5)	0.77 (0.28–2.18)	
Yes	11 (25.0)	8 (20.5)	1.00 (reference)	
BMI, kg/m^2 ^				0.319
≤25	24 (54.5)	17 (43.6)	1.55 (0.65–3.70)	
>25	20 (45.5)	22 (56.4)	1.00 (reference)	
Pleural effusions				0.001
No	37 (84.1)	18 (46.2)	6.17 (2.21–17.17)	
Yes	7 (15.9)	21 (53.8)	1.00 (reference)	
Ascites				0.003
No	29 (65.9)	13 (33.3)	3.87 (1.55–9.63)	
Yes	15 (34.1)	26 (66.7)	1.00 (reference)	
Tumor bilaterality				0.001
Unilateral	34 (77.3)	14 (35.9)	6.07 (2.32–15.89)	
Bilateral	10 (22.7)	25 (64.1)	1.00 (reference)	
Largest tumor size, mm				0.037
<60	27 (61.4)	15 (38.5)	4.44 (1.30–15.24)	
≥60	17 (38.6)	24 (61.5)	1.00 (reference)	
Lymph nodes				0.012
No	40 (90.9)	27 (69.2)	1.55 (0.65–3.70)	
Yes	4 (9.1)	12 (30.8)	1.00 (reference)	
Omental caking				0.003
No	37 (84.1)	21 (53.8)	4.53 (1.63–12.62)	
Yes	7 (15.9)	18 (46.2)	1.00 (reference)	
Peritoneal thickening				0.001
No	37 (79.5)	13 (35.9)	10.57 (3.71–30.11)	
Yes	7 (20.5)	26 (64.1)	1.00 (reference)	
Extrapelvic tumor >2 cm				0.001
No	33 (75.0)	15 (38.5)	4.80 (1.88–12.28)	
Yes	11 (25.0)	24 (61.5)	1.00 (reference)	
Serum CA-125 levels, U/mL				0.001
≤370	33 (75.0)	9 (23.1)	10.00 (3.64–27.46)	
>370	11 (25.0)	30 (76.9)	1.00 (reference)	
Hemoglobin levels, g/dL				0.096
≤10.5	19 (43.2)	24 (61.5)	0.48 (0.20 – 1.14)	
>10.5	25 (56.8)	15 (38.5)	1.00 (reference)	
White cells count, ×10^9^/L				0.429
≤6.5	21 (47.7)	22 (56.4)	0.71 (0.30–1.68)	
>6.5	23 (52.3)	17 (43.6)	1.00 (reference)	
Platelet count, ×10^9^/L				0.907
≤333	22 (50.0)	20 (51.3)	3.87 (1.55–9.63)	
>333	22 (50.0)	19 (48.7)	1.00 (reference)	

The article "Preoperative Predictors of Optimal Tumor Resectability in Patients With Epithelial Ovarian Cancer" was published in 2022. Journal: Cureus.

**Table 3:** Multivariate analyses of preoperative predictors of optimal surgical resection in epithelial ovarian cancer (n = 83). CA-125: cancer antigen-125; CI: confidence interval; OR: odds ratio

Characteristics	Category	Multivariate	
		Adjusted OR (95% CI)	P-value
Ascites	No vs. yes	1.83 (0.38–8.79)	0.452
Pleural effusions	No vs. yes	5.60 (1.32–23.71)	0.019
Tumor bilaterality	Unilateral vs. bilateral	2.02 (0.43–9.52)	0.374
Largest tumor size	<60 vs. ≥60 mm	2.86 (0.74–11.06)	0.127
Omental caking	No vs. yes	0.59 (0.12–2.84)	0.506
Peritoneal thickening	No vs. yes	2.76 (0.51–14.92)	0.237
Extrapelvic tumor >2 cm	No vs. yes	2.45 (0.51–11.68)	0.262
Retroperitoneal lymph nodes	Absent vs. present	3.42 (0.42–28.16)	0.253
Serum CA-25 levels	≤370 vs. >370 U/mL	6.80 (1.19–38.79)	0.031
Hemoglobin concentration	≤10.5 vs. >10.5 g/dL	0.99 (0.27–3.63)	0.984

Furthermore, as shown in the univariate analyses reported in Table 4, the absence of preexisting comorbidity (P = 0.088) and serum CA-125 levels (P = 0.005) together with the absence of radiological evidence of pleural effusion (P = 0.007), tumor bilaterality (P = 0.037), significant preoperative tumor size (P = 0.059), peritoneal thickening (P = 0.001), and retroperitoneal lymph nodes (P = 0.001) were the likely predictors of OTR in patients with advanced EOC. On multivariate analyses, the absence of medical comorbidities (OR = 18.21; 95% CI = 2.40, 38.10; P = 0.005) and radiological absence of pleural effusions (OR = 13.75; 95% CI = 1.80, 24.85; P = 0.011) and retroperitoneal lymph nodes (OR = 11.95; 95% CI = 1.35, 16.07; P = 0.026) were independently associated with OTR in patients with FIGO stage III and IV disease during PDS.

**Table 4:** Univariate and multivariate analyses of preoperative predictors of optimal surgical resection in advanced epithelial ovarian cancer (n = 61). BMI: body mass index; CA-125: cancer antigen-125; OR: odds ratio

Characteristics	Category	Optimal tumor resection		
		Univariate	Multivariate	
		P-value	Adjusted OR (95% CI)	P-value
Comorbidity	No vs. yes	0.045	18.21 (2.40–38.10)	0.005
BMI, kg/m^2^	≤25 vs. >25	0.923	-	-
Ascites	No vs. yes	0.554	-	-
Pleural effusions	No vs. yes	0.007	13.75 (1.80–24.85)	0.011
Tumor bilaterality	Unilateral vs. bilateral	0.037	2.37 (0.44–12.87)	0.319
Largest tumor size, mm	<60 vs. ≥60	0.090	4.75 (0.84–26.91)	0.078
Omental caking	No vs. yes	0.147	-	-
Peritoneal thickening	No vs. yes	0.001	6.21 (0.74–52.13)	0.093
Extrapelvic tumor >2 cm	No vs. yes	0.225	-	-
Retroperitoneal lymph nodes	Absent vs. present	0.001	11.95 (1.35–16.07)	0.026
Serum CA-25 levels	≤370 vs. >370 U/mL	0.005	4.32 (0.55–34.04)	0.165
Hemoglobin concentration, g/dL	≤10.5 vs. >10.5	0.225	-	-
White cell count, ×10^9^/L	≤6.5 vs. >6.5	0.411	-	-
Platelet count, ×10^9^/L	≤333 vs. >333	0.662	-	-

The article "Preoperative Predictors of Optimal Tumor Resectability in Patients With Epithelial Ovarian Cancer" was published in 2022. Journal: Cureus.

## Discussion

This study investigated the preoperative predictors of optimal PDS in patients with EOC in Lagos, Nigeria. This was based on the report of a paradigm shift by Horowitz et al. [11] who reported that if an optimal surgical outcome is difficult to attain with upfront surgical debulking, then the use of NACT followed by IDS may be superior to PDS, especially in patients with advanced-stage disease. In this study, we found that the radiological absence of pleural effusion and serum CA-125 levels of ≤370 U/mL were the only independent predictors of OTR in patients with EOC. Furthermore, in patients with advanced-stage III and IV disease, the absence of preexisting comorbidity, pleural effusions (on chest imaging), and retroperitoneal lymph nodes were the independent predictors of OTR.

The overall rate of OTR in this study (53.0%) is higher than the rates reported in previous studies by Kim et al. (40.0%) [12], Rutten et al. (46.4%), [8], and Gerestein et al. (45.0%) [13]. However, the rate of OTR recorded in patients with advanced EOC only (36.1%) in our study is similar to the rates reported in previous studies that included only patients with advanced (FIGO stage III and IV) disease. Only a few studies have reported on the predictors of optimal surgical debulking in patients with EOC, most of which relied on radiologic predictors [14-17], unlike our study that used patients’ clinical parameters such as the presence of medical comorbidities, BMI, hematologic, and biochemical markers, in addition to the radiologic evidence of pleural effusion, ascites, tumor bilaterality, largest tumor size, retroperitoneal lymphadenopathy, omental cake, significant extrapelvic tumor, and peritoneal thickening. Our results showed that the presence of pleural effusions on preoperative imaging increased the risk of suboptimal debulking by up to 14 times in patients with advanced EOC. In patients with OC, moderate-to-large pleural effusions have been reported to be more likely to be malignant [18], a finding that automatically upstages the disease to at least FIGO stage IV [19], thus suggesting the increased tendency of having a residual disease after PDS [20].

The most commonly studied biomarker for EOC is serum CA-125 level [21]. Chi et al. [22] in 2000 and Kang et al. [9] in 2010 reported that preoperative serum CA-125 levels greater than 500 U/mL were strongly associated with suboptimal surgical debulking in patients with advanced EOC. This was further corroborated by the findings of our study where a lower serum CA-125 cut-off level of 370 U/mL was associated with increased odds of OTR. The most appropriate cut-off of CA-125 remains somewhat controversial, and a future validation study can help confirm the most appropriate value. We reported a significant reduction in the rate of OTR among advanced EOC patients with coexisting medical morbidities, which may be explained by the reduced tendency of these patients to tolerate prolonged anesthesia and extensive tumor debulking with a resultant decrease in available surgical time for optimal resection of all visible tumors.

The article "Preoperative Predictors of Optimal Tumor Resectability in Patients With Epithelial Ovarian Cancer" was published in 2022. Journal: Cureus.

Metastasis via retroperitoneal lymph nodes is one of the main pathways of OC spread at a rate that is as high as 44-53% in advanced OC [23,24]. Only 19.30% of patients in our study had any radiologic evidence of enlarged retroperitoneal lymph nodes, but the rate of microscopic lymph node metastasis, even though not reported, could be much higher. Retroperitoneal lymph node enlargement on radiologic imaging was reported to be a predictor of OTR in our study. This corroborated the findings of Bristow et al. [25] and Suidan et al. [26] who reported suprarenal para-aortic lymph node enlargement (≥1 cm) as one of the most important predictive factors for suboptimal debulking in patients with advanced OC.

In this study, the rate of successful OTR was 65.9% in patients with no visible ascites on imaging and 34.1% in patients with EOC and ascites. This is, however, in contrast to the study by Randle et al. [27] who reported that the rate of complete cytoreductive surgery in patients with OC and malignant ascites remained 100%. Massive ascites may affect the respiratory and circulatory functions of patients with subsequent decreased ability to withstand prolonged anesthesia and extensive surgical resection [28]. Our study is also corroborated by the findings from other previous studies [29,30] that reported ascites as one of the predictors of suboptimal surgical debulking in OC patients. However, no independent association was recorded between ascites and OTR in the final multivariate models used in our study.

A significant strength of this study is the initial review of all cases and the performance of debulking surgeries in a multidisciplinary team setting involving the gynecologic oncologist, general/colorectal surgeon, and urologist, with the reduction in the influence of this factor on the oncologic outcome (OTR) being examined in the study. However, the study has a few limitations. First, because this was a single-center retrospective study, the findings cannot be generalizable to other gynecologic oncology units or centers in the country. Second, the number of patients who were eligible for PDS during the review period was relatively small, limiting the in-depth analysis, conclusions, and generalizability of the study findings. The important influence of the cadre and experience of the lead surgeons on the OTR rate was not assessed as the available data in the review was not sufficient to examine this. We intend to investigate this in future research work. In addition, this study only included patients who had PDS followed by adjuvant chemotherapy with the exclusion of patients treated with NACT who could have had a high proportion of the authors’ identification predictors that could have a significant impact on the study endpoints. Finally, the lack of data on patients’ performance status, which is evidence of patients’ cardiovascular and respiratory stability, could significantly influence the extent of the upfront debulking surgery and act as an important confounding factor.

The article "Preoperative Predictors of Optimal Tumor Resectability in Patients With Epithelial Ovarian Cancer" was published in 2022. Journal: Cureus.

## Conclusions

It is important to predict patients with advanced EOC who may benefit from upfront primary surgical debulking with the use of certain preoperative clinical and radiological parameters to reduce the surgical morbidity and improve the oncologic outcome of these patients. In this study, we demonstrated that having no preexisting comorbidity, serum CA-125 of ≤370 U/mL, and absence of radiologic evidence of large pleural effusions and enlarged retroperitoneal lymph nodes were independent predictors of OTR. However, this is a pilot study among women with EOC in Nigeria. The preliminary data generated will be further tested in a future validation study.
